RETRACTED

# Unreferenced English articles’ translation quality-oriented automatic evaluation technology using sparse autoencoder under the background of deep learning

**DOI:** 10.1371/journal.pone.0270308

**Published:** 2022-07-13

**Authors:** Hanhui Li, Jie Deng

**Affiliations:** 1 School of Foreign Languages, Fuzhou University of International Studies and Trade, Fuzhou City, China; 2 Graduate School, Angeles University Foundation, Angeles City, Philippines; 3 Rockchip Electronics Co., Ltd., Fuzhou City, China; University of Bonab, ISLAMIC REPUBLIC OF IRAN

## Abstract

Currently, both manual and automatic evaluation technology can evaluate the translation quality of unreferenced English articles, playing a particular role in detecting translation results. Still, their deficiency is the lack of a close or noticeable relationship between evaluation time and evaluation theory. Thereupon, to realize the automatic Translation Quality Assessment (TQA) of unreferenced English articles, this paper proposes an automatic TQA model based on Sparse AutoEncoder (SAE) under the background of Deep Learning (DL). Meanwhile, the DL-based information extraction method employs AutoEncoder (AE) in the bilingual words’ unsupervised learning stage to reconstruct the translation language vector features. Then, it imports the translation information of unreferenced English articles into Bilingual words and optimizes the extraction effect of language vector features. Meantime, the translation language vector feature is introduced into the automatic DL-based TQA. The experimental findings corroborate that when the number of sentences increases, the number of actual translation errors and the evaluation scores of the proposed model increase, but the Bilingual Evaluation Understudy (BLEU) score is not significantly affected. When the number of sentences increases from 1,000 to 6,000, the BLEU increases from 96 to 98, which shows that the proposed model has good performance. Finally, the proposed model can realize the high-precision TQA of unreferenced English articles.

## Introduction

Human society has seen progress and development through cultural exchange and collision. As the main carrier of different cultural exchanges, the translation between different languages is the key to multicultural exchanges. Therefore, translation technology is indispensable in disseminating cultural information [1, 2]. In the era of global economic integration, translation technology has become one of the industries attracting worldwide attention, which has promoted the development of the country’s foreign economy. Machine Translation (MT) tasks began in the 1950s. Since the 1990s, MT has entered a period of rapid development thanks to soaring computing performance, storage capacity, and more available corpus. Meanwhile, with the extensive development of the MT system, MT evaluation has also risen sharply. It has become an active research field and a hot topic for discussion [3–5]. Scholars try to understand how well MT results are and whether they are eligible to replace manual translation. At the same time, by evaluating MT, researchers can intuitively demonstrate the MT system’s performance for optimization and fine-tune. Since manual labor demands considerable time and money, the automatic Translation Quality Assessment (TQA) method came into being. Most commonly, calculating the similarity between the MT results and manual works can improve the MT system performance. Besides, the comparison can partially reflect the quality of MT works [6].

RETRACTED

In the current MT-oriented Translation Quality Assessment (TQA), the automatic TQA technology for artificial translation of reference-based English articles is widely used. Nevertheless, the evaluation results depend entirely on the given reference articles, which focus on reflecting the performance of the Machine Translation Systems (MTSs). However, translation references are not necessarily correct and practical [7]. Some scholars have also applied fuzzy logic systems and Deep Learning (DL) technology to non-artificial translation reference-based (unreferenced) English articles translation. They find that although it can roughly express the meaning of the article, there are still some defects in the "faithfulness, expressiveness, and elegance" of the translated language. If these technologies are to be applied to translation, they need continuous improvement and optimization [8]. Therefore, more and more researchers have begun to study the new MT-oriented TQA technology for unreferenced English article translation. Accordingly, this paper compares the unreferenced English articles-oriented and referenced English articles-oriented TQA. It finds that the unreferenced English articles-oriented TQA poses no standard restrictions on reference articles and can be applied in the research stage and be popularized in practical applications [9, 10]. Apparently, such an unreferenced English articles-oriented TQA is more practical and has more research value.

At present, the unreferenced English articles-oriented TQA technique is still in the early stage of development. It is not technologically mature, but there is room for growth and progress in practical applications. In summary, the current research shows that China has not paid enough attention to the TQA technology of unreferenced English articles compared with European and American countries. Accordingly, under the background of Deep Learning (DL), this paper proposes an automatic TQA model for unreferenced English articles based on Sparse AutoEncoder (SAE): the DL algorithm is applied to TQA and Feature Extraction (FE) to realize the high-precision TQA for MT.

RETRACTED

## Automatic TQA model

### SAE

#### (1) Back Propagation (BP) algorithm

BPNN belongs to a nonlinear intelligent learning system. Through the simulation of the human brain information processing mode and back-propagation according to the error, the weight and threshold of the BPNN are continuously adjusted, and the Gradient Descent Method (GDM) is used to complete the calculation [11–13]. Adjusting the weight and threshold can minimize the error between the corresponding expected and the actual output, making the actual output closer to the expected value and improving the network learning adaptability.

The forward-propagation process and the back-propagation process of the BPNN algorithm constitute the common process of error propagation. In the forward-propagation process of the signal, it is necessary to provide input samples to each neuron of the input layer, calculate the net input and output of the output layer and each hidden layer, and then calculate the prediction results of the neural network [14, 15]. If there is a large error between the calculated prediction result and the expected output, the back-propagation of the error is started. In the process of error back-propagation, it is necessary to input the error back into the output layer, back-propagate the error, and update the weight according to the error of each layer. Simultaneously, the weight will be updated and adjusted continuously. Until the learning process reaches the preset number of iterations or the output error is less than the specified threshold, the learning process is terminated [16, 17].

Fig 1 draws the structure of BPNN, including the input layer, hidden layer, and output layer. The hidden layers can be one or multiple, each with several nodes.

**Fig 1:** BPNN structure.

In the process of forwarding calculation, when the data in the input layer of BP NN is *x*_1_, *x*_2_, *x*_3_,…,*x*_*n*_, the input of each neuron in the hidden layer is calculated by Eq (1):

$$h_{i}=\sum_{j=1}^{n}\;w_{ij}x_{j}+p_{i}(i=1,2,\ldots ,m)$$ (1)

In Eq (1), *n*, *m*—the number of neurons in the input layer and hidden layer. *w*_*ij*_—connection weight between *j* neuron in the input layer and *i* neuron in the hidden layer. *p*_*i*_—the threshold of neurons in hidden layer *i*. *h*_*i*_—input of *i* neuron in the hidden layer.

The hidden layer adopts the Sigmoid function as the Activation Function (AF) of the neurons, so the output of neurons in the hidden layer can be expressed by Eq (2):

$$o_{i}=f(h_{i})(i=1,2,\ldots ,m)$$ (2)

In Eq (2), the AF $f(x)=\frac{1}{1+e^{-x}}$. The output layer adopts the identity function as the AF of neurons, and the threshold is 0. Then the output of each neuron in the output layer can be expressed by Eq (3):

$$y_{k}=\sum_{i=1}^{m}\;v_{ki}o_{i}(k=1,2,\ldots ,l)$$ (3)

In Eq (3), *v*_*ki*_—connection weight between *i* neuron in the hidden layer and *k* neuron in the output layer. *l*—the number of neurons in the output layer.

RETRACTED

The connection weights between the neurons in the input layer and the hidden layer form the weight vector W. After the weight vector *W* is determined, the output can be calculated according to the input of the neural network.

The learning samples of the back-propagation are (*x*_1*r*_, *x*_2*r*_,…,*x*_*nr*_; *t*_*kr*_), *r* = 1,2,…,*r*, where *r* is the number of samples. After the weight vector *W* is given, the actual output *y*_*kr*_ of the neural network can be calculated, and the error functions of output error and learning sample *r* are defined as $d_{kr}=t_{kr}-y_{kr},\;e_{r}=\frac{1}{2}\sum_{k=1}^{r}\;{\left(t_{kr}-y_{kr}\right)}^{2}$.

The value of weight vector *W* is random in the initial case, so the actual calculated output *y*_*kr*_ of the network is not high. After the neuron number *m* is determined in the hidden layer, the error *d*_*kr*_ can be reduced by adjusting the W. Back-propagation is along the function *e*_*r*_ and adjusts the weight vector with the negative gradient direction [18–20]. Then, the correction value of weight vector *W* is set as Δ*W* and calculated as $\Delta W=-\eta \frac{\partial e_{r}}{\partial W}$, where *η* is the learning rate (0–1). Eqs (4)–(8) are obtained through calculation:

$$\Delta W=\eta \sum_{k=1}^{l}\;d_{kr}\frac{\partial y_{kr}}{\partial W}$$ (4)

$$\Delta W=(\Delta v_{ki},\Delta p_{i},\Delta w_{ij})$$ (5)

$$\Delta v_{ki}=\eta d_{kr}o_{ir}$$ (6)

$$\Delta p_{i}=\eta o_{ir}(1-o_{ir})\sum_{k=1}^{l}\;d_{kr}v_{ki}$$ (7)

$$\Delta W=\eta o_{ir}(1-o_{ir})x_{jr}\sum_{k=1}^{l}\;d_{kr}v_{ki}$$ (8)

Next, *ΔW* can be calculated by Eqs (4)–(8). Then, the weight vector is modified according to *W* = *W*+*ΔW* [21].

#### (2) Auto Encoder (AE) algorithm

AE is a typical three-layer neural network structure proposed by Rumelhart. The network structure includes an input layer, an output layer, and a hidden layer. The dimension of the output and the input layer is both n, and the dimension of the hidden layer is m [22, 23]. Fig 2 gives the structure of an AE:

**Fig 2:** AE network structure.

The encoding process refers to the process from the input layer to the hidden layer, and the decoding process refers to the process from the hidden layer to the output layer. If the encoding function and decoding function are set to *f* and *g*, respectively, Eqs (9) and (10) can be obtained:

$$h=f(x)=s_{f}(wx+p)$$ (9)

$$y=g(h)=s_{g}(\tilde{w}h+q)$$ (10)

In Eqs (9) and (10), *s*_*f*_—AF of the encoder, usually Sigmoid function, calculated by $f(x)=\frac{1}{1+e^{-x}}$. *s*_*g*_—AF of decoder, usually taking identity function or Sigmoid function. *w*—weight matrix between the hidden layer and input layer. $\tilde{w}$—the weight matrix between the output layer and the hidden layer, and $\tilde{w}=w^{⊤}.\;\theta =\{w,p,q\}$ is the parameters of AE.

RETRACTED

The output *Y* of the output layer can be regarded as the predicted value of the input *X* of the input layer. AE can use the BP algorithm to adjust the neural network parameter. When the error between the input *X* and the output *Y* is within the acceptable range, AE retains most of the information of the original input data. At this time, the training process of the AE neural network is completed [24]. The proximity between *X* and *Y* is defined as the error function *L*(*x*,*y*). Then, when the AF of the decoder is an identity function, *L*(*x*,*y*) = ‖*x*−*y*‖^2^ can be obtained.

When the AF of the decoder is Sigmoid function, Eq (11) can be obtained:

$$L(x,y)=-\sum_{i=1}^{n}\;[x_{i}logy_{i}+(1-x_{i})log(1-y_{i})]$$ (11)

When $S={\left\{X^{\left(i\right)}\right\}}_{i=1}^{N}$ is a given training sample set, the overall loss function of AE can be expressed by Eq (12):

$$J_{AE}(\theta )=\sum_{x\in S}\;L(x,g(f(x)))$$ (12)

Finally, GDM is used to calculate the minimum of iteratively *J*_*AE*_(*θ*) to determine the AE parameters. Then, the training process of AE can be ended [25, 26].

#### (3) SAE

SAE has certain requirements for the sparsity of neuron activation degree in the hidden layer. When the input data is *x*, the activation degree of neuron *j* in the hidden layer can be expressed as *h*_*j*_(*x*), and then the Eq (13) can be obtained:

$${\hat{\rho }}_{j}=\frac{1}{N}h_{j}(x^{\left(i\right)})$$ (13)

In Eq (13), ${\hat{\rho }}_{j}$–average activation of the hidden layer neuron *j* on the sample set $S={\left\{X^{\left(i\right)}\right\}}_{i=1}^{N}$. Thus, to make the sparsity of neurons in the hidden layer meet the constraints, ${\hat{\rho }}_{j}=\rho ,\;(j=1,2,\ldots ,m)$, where *ρ* is a small sparsity parameter (*ρ* = 0.05). If *ρ* and ${\hat{\rho }}_{j}$ are too far apart, *KL*(Kullback-Leibler) divergence shall be used to adjust it. The function of $KL(\rho ∥{\hat{\rho }}_{j})$ is defined as in Eq (14):

$$KL(\rho ∥{\hat{\rho }}_{j})=\rho *log\frac{\rho }{{\hat{\rho }}_{j}}+(1-\rho )*log\frac{1-\rho }{1-{\hat{\rho }}_{j}}$$ (14)

The greater the difference between *ρ* and ${\hat{\rho }}_{j}$, the larger $KL(\rho ∥{\hat{\rho }}_{j})$ will be. When $\rho ={\hat{\rho }}_{j}$, the function value reaches the minimum [27–30]. Therefore, if $KL(\rho ∥{\hat{\rho }}_{j})$ is added to the AE loss function, then *ρ* and ${\hat{\rho }}_{j}$ get as close as possible when $\rho ={\hat{\rho }}_{j}$. Accordingly, the loss function of SAE can be obtained, as in Eq (15):

$$J_{SAE}(\theta )=\sum_{x\in S}\;L(x,g(f(x)))+\beta \sum_{j=1}^{m}\;KL(\rho ∥{\hat{\rho }}_{j})$$ (15)

In Eq (15), *β*—the weight coefficient to control the sparsity penalty. After the loss function *J*_*SAE*_(*θ*) is minimized, the parameter *θ* can be obtained.

RETRACTED

The previous section has expounded on the relevant theories of SAE and AE. Their difference is explained as follows. The SAE can be obtained by adding the corresponding regular restriction on the basis of AE. Comparing the two encoders reveals that the SAE can impose constraints on the loss function. SAE reflects the unique statistical characteristics of the training data set rather than simply acting as an identity function. By training the data in this way, a model can be designed to learn useful features. Finally, numerous training parameters will complicate the training process. The dimension of training output is much higher than that of input. This will produce much redundant data information. Adding SAE can add value to the learned features, which is also in line with the characteristics of the sparse response of human brain neurons.

AE can reconstruct the input data. The middle layer of an AE is the feature expression of the input data. The stacked AE method removes the output layer of the previous AE and imports the feature map of the hidden layer to the next AE. Accordingly, the Deep Neural Network (DNN) structure of the Stacked AE can be formed. A Softmax classifier is connected at the end of the Stacked AE structure for classification operation. The Stacked AE DNN is trained in layers, including the final classifier. Each layer is trained by the back-propagation algorithm. The structure of DNN constructed based on sparse edge noise reduction AE is demonstrated in Fig 3:

**Fig 3:** Network structure.

After the DNN model of AE based on sparse edge noise reduction is constructed, the layer-wise greedy training algorithm is used for training. It mainly includes two stages: pre-training and fine-tuning. The algorithm flow is listed in Table 1:

**Table 1:** Algorithm flow chart.

Input:	
Train:	The training set is used to train the network model and determine its parameters.
Valid:	The validation set is used to determine the optimal network model.
Test:	The test set tests the classification ability of the network model with different classes.
pretrain_lr	Pre-training learning rate.
finetune_lr	Fine-tuning learning rate.
pretrain_epoches:	Pre-training number of iterations.
training_epoches:	The maximum iterations in fine-tuning phase
Rho:	Sparsity parameter of SAE
Beta:	Control the weight coefficient of the sparsity penalty term
Output:	
validation_score:	Validation set error rate
test performance:	Test set error rate
Method:	
1)	A two-layer stacking network model is constructed to determine the size of the block minibatch of the three data sets.
2)	Through the network model constructed in (1), the calculation method of the pre-training loss function of the model is obtained.
3)	For hidden layer *i* the network model:
	For an epoch in pretrain_epoches:
	For a batch_index in minibatch:
	Call the loss function calculation method obtained in (2) to calculate the loss after each hidden layer is encoded and decoded. Use the BP algorithm to adjust the model parameters.
4)	Output the average loss of an epoch in each layer.
5)	The model parameters are determined through the network model constructed in (1). The calculation method of the fine-tuning stage of the model is obtained.
6)	Do
7)	Keep iterating to find the best_validation_loss of this_validation_loss in the test set. Update best_validation_loss.
8)	When best_validation_loss is updated, calculate the error rate in the test
9)	Until iteration epoch>training_epoches or done_looping = True
10)	Output validation_score and test performance

The algorithm is coded below:

from sklearn.datasets import make_blobs

from tensorflow.keras.layers import Dense

from tensorflow.keras.models import Sequential

from tensorflow.keras.optimizers import SGD

from tensorflow.keras.utils import to_categorical

import matplotlib.pyplot as plt

plt.rcParams[’figure.dpi’] = 200

RETRACTED

# 1. Data preparation

def prepare_data():

    # Sample generation

    X, y = make_blobs(n_samples = 1000, centers = 3, n_features = 2, cluster_std = 2, random_state = 2)

    # one-hot coding

    y = to_categorical(y) # tf.keras.utils.to_categorical

    # Division of training set and verification set (test set)

    n_train = 500

    trainX, testX = X[:n_train,:], X[n_train:,:]

    trainy, testy = y[:n_train], y[n_train:]

    return trainX, testX, trainy, testy

# 2. Model definition

def get_base_model(trainX, trainy):

    # Model definition

    model = Sequential()

    model.add(Dense(10, input_dim = 2, activation = ’relu’, kernel_initializer = ’he_uniform’))

    model.add(Dense(3, activation = ’softmax’))

    # Model compilation

    opt = SGD(lr = 0.01, momentum = 0.9)

    model.compile(loss = ’categorical_crossentropy’, optimizer = opt, metrics = [’accuracy’])

    # Model training

    model.fit(trainX, trainy, epochs = 100, verbose = 0)

    return model

# 3. Evaluate model

def evaluate_model(model, trainX, testX, trainy, testy):

    _, train_acc = model.evaluate(trainX, trainy, verbose = 0)

    _, test_acc = model.evaluate(testX, testy, verbose = 0)

    return train_acc, test_acc

# 4. Greedy layer-by-layer pre training configuration

def add_layer(model, trainX, trainy):

    # Keep the output layer to add a new hidden layer

    output_layer = model.layers[–1]

    model.pop()

    # Set the previous layer as untrainable to ensure that the weight is not updated

    for layer in model.layers:

    layer.trainable = False

    # Add a hidden layer with the same configuration as the first layer of the basic model

    model.add(Dense(10, activation = ’relu’, kernel_initializer = ’he_uniform’))

    model.add(output_layer)

    # Model training

    model.fit(trainX, trainy, epochs = 100, verbose = 0)

# Data preparation

trainX, testX, trainy, testy = prepare_data()

# Basic model

model = get_base_model(trainX, trainy)

# Create a dictionary to save the accuracy of different hidden layer models

scores = {}

# Training and evaluation

train_acc, test_acc = evaluate_model(model, trainX, testX, trainy, testy)

# Print accuracy

print(’> layers = %d, train = %.3f, test = %.3f’ % (len(model.layers), train_acc, test_acc))

# Save accuracy

scores[len(model.layers)] = (train_acc, test_acc)

n_layers = 10

for i in range(n_layers):

    # Add hidden layer

    add_layer(model, trainX, trainy)

    # Model evaluation

    train_acc, test_acc = evaluate_model(model, trainX, testX, trainy, testy)

    print(’> layers = %d, train = %.3f, test = %.3f’ % (len(model.layers), train_acc, test_acc))

    # The accuracy is stored in the dictionary to facilitate drawing

    scores[len(model.layers)] = (train_acc, test_acc)

plt.plot(list(scores.keys()), [scores[k][0] for k in scores.keys()], label = ’train’, marker = ’.’)

plt.plot(list(scores.keys()), [scores[k][1] for k in scores.keys()], label = ’test’, marker = ’.’)

plt.legend()

plt.show()

The core idea of the layer-by-layer greedy algorithm is to construct an optimal solution step by step. Each step makes an optimal decision under certain standards, and the decision made in each step cannot be changed in the next steps. For example, for the loading of containers, load the containers onto the arrival ship step by step, and load one container step by step. Each step determines which container to load. The greedy criterion for making decisions is to select the container with the smallest weight from the remaining containers to ensure the minimum total weight of the selected container. The cargo ship can load more containers with the maximum capacity. Additionally, the knapsack problem also involves a layer-by-layer greedy algorithm. For a knapsack with *n* items and a capacity of *c*, the packed items are selected from *n* items. The weight of article *i* is *w*_*i*_. The value is *p*_*i*_. A feasible knapsack loading means that the total weight of the packed items does not exceed the capacity of the knapsack. An optimal backpack load refers to the feasible backpack load with the highest total value of goods. The backpack problem can be described by Eq (16)–(17):

$$max\sum_{i=1}^{n}\;p_{i}x_{i}$$ (16)

The constraints are:

$$\sum_{i=1}^{n}\;w_{i}x_{i}⩽c\;\mathrm{and}\;x_{i}\in \{0,1\}1⩽i⩽n$$ (17)

In Eqs (16)–(17), the value of *x*_*i*_ must be calculated. *x*_*i*_ = 1 means that the item *i* is loaded into the backpack. Otherwise, *x*_*i*_ = 0 means item *i* is not loaded into the backpack.

RETRACTED

### Translation language information extraction

This section sets the hyperparameter as the translation quality of unreferenced English articles. The language information is fused through the automatic translation language-oriented information extraction method. In the context of DL, the learning and training process of language information extraction method for translation of English articles without reference consists of two stages: the supervised learning stage and the unsupervised learning stage. In the unsupervised learning stage, the AE is mainly used to learn and train the words of the Source Language (SL) and Target Language (TL), and then the bilingual semantic features of the two languages are obtained. In the supervised learning stage, to optimize the extraction effect of language vector features, it is necessary to import the standard information of Natural Language (NL) corpora into bilingual words to realize the fine-tuning of bilingual semantic features [31, 32].

The unsupervised learning stage takes the training corpus of SL A and TL B as the learning objects. Fig 4 demonstrates the learning diagram:

**Fig 4:** Learning diagram. a: SL A vector reconstruction; b: TL B vector reconstruction.

The unsupervised learning stage learns the training corpus of source language A and translation results of target language B. Translation result of B must not be entirely consistent with A. Then, the automatic MT system is trained by vector A (*Y*_*E*_) and vector B (*Y*_*C*_) to obtain the bilingual aligned sample pairs (*Y*_*E*_, *Y*_*C*_). (*Y*_*E*_, *Y*_*C*_) represents a bilingual word. Based on this, noise reduction AE is used to learn the bilingual word (*Y*_*E*_, *Y*_*C*_) unsupervised to reconstruct the new vector A and vector B for vector B in sample *y* are reconstructed. Finally, the language vector features in the automatic MT sample are obtained.

RETRACTED

Next, the two NLs are learned through the AE to optimize the unsupervised learning process’s reliability. Before reconstructing the vectors *A*, *B* in sample *y*, a certain degree of noise is introduced into the sample pair (*Y*_*E*_, *Y*_*C*_) to $\left({\bar{Y}}_{E},\;{\bar{Y}}_{C}\right)$ vector. The AE can implicitly express *k*_*E*_, *k*_*C*_ of the two NLs *A*, *B* through the Sigmoid AF, as demonstrated in Eqs (18) (19):

$$k_{E}=g_{\theta }({\bar{Y}}_{E})=r(V_{E}\cdot {\bar{Y}}_{E}+\beta )$$ (18)

$$k_{C}=g_{\theta }({\bar{Y}}_{C})=r(V_{C}\cdot {\bar{Y}}_{C}+\beta )$$ (19)

In Eqs (18) and (19), *g*_*θ*_—coding function; *r*—AF; *V*_*E*_, *V*_*C*_—translation matrix parameters, which are bilingual words with their unique language characteristics; ${\bar{Y}}_{E},\;{\bar{Y}}_{C}$—Bilingual words; *β*—bias. Since *k*_*E*_, *k*_*C*_ have the same dimension, *β* is shared by *A*, *B*.

After *k*_*E*_, *k*_*C*_ is obtained, AE decodes the implicit expressions of A and B, and *k*_*E*_ is decoded to obtain the reconstructed vector ${\hat{y}}_{c}$ of TL and reconstruction vector y of SL ${\hat{y}}_{E}$. Eqs (20) (21) specify the results:

$${\hat{y}}_{C}=g_{\theta }(k_{C})=r(V_{C}\cdot k_{C}+d_{C})$$ (20)

$${\hat{y}}_{E}=g_{\theta }(k_{E})=r(V_{E}\cdot k_{E}+d_{E})$$ (21)

In Eqs (20) and (21), *g*_*θ*_—decoding function; *d*_*C*_, *d*_*E*_—decoder bias of language.

The decoding method of implicit *k*_*E*_ is the same as the decoding steps *k*_*C*_. Then, implicit *k*_*E*_ can be decoded to obtain ${\hat{y}}_{E}$, and the implicit *k*_*C*_ can be decoded to obtain ${\hat{y}}_{C}$.

This kind of encoding and decoding form can reconstruct one NL to get the vector of another NL. It can also be transformed into the vector of the SL. However, due to the difference in information between the two NLs, some errors will be caused in reconstruction. Accordingly, *Y*_*E*_ is reconstructed to obtain the SL vector and the corresponding error *p*(*Y*_*E*_). Meanwhile, *Y*_*C*_ is reconstructed to obtain the original vector and the corresponding error *p*(*Y*_*C*_). Afterward, *Y*_*C*_ is reconstructed to obtain the SL vector *Y*_*E*_ and the corresponding error *p*(*Y*_*C*_, *Y*_*E*_). (*Y*_*E*_, *Y*_*C*_) is reconstructed to obtain the error of the original vector pair $p[(Y_{C},\;Y_{E}),\;({\hat{y}}_{C},\;{\hat{y}}_{E})]$. Lastly, the reconstruction error of the sample pair (*Y*_*E*_, *Y*_*C*_) is set as the cross-entropy, and the sum of five kinds of reconstruction errors *p*(*Y*_*E*_), *p*(*Y*_*C*_), *p*(*Y*_*E*_, *Y*_*C*_), *p*(*Y*_*C*_, *Y*_*E*_), $p[(Y_{C},\;Y_{E}),\;({\hat{y}}_{C},\;{\hat{y}}_{E})]$ is set as the loss function in the unsupervised learning stage [33–35].

RETRACTED

The decoding function in the unsupervised learning process is set as *g*_*θ*_ = {*V*_*E*_, *V*_*C*_, *d*_*E*_, *d*_*C*_}, which the GDM updates to minimize the loss function, and *V*_*E*_, *V*_*C*_ is obtained after training.

### TQA of unreferenced English articles

The DL-based unreferenced English articles-oriented TQA model is composed of one regression layer, one hidden layer, and three visual layers, which are represented by *t*_1_, *t*_2_, *t*_3_ respectively. The trained *V*_*E*_, *V*_*C*_ will be input to the visual layer, the three hidden layers contain 100 nodes, and the regression layer contains one node and outputs the results. The Joint Probability Distribution (JPD) of the hidden layer and visible layer is calculated by Eq (22):

$$Q_{\theta }=Q(t_{1})\cdot Q(t_{2})\cdot Q(t_{3})$$ (22)

In Eq (22), *Q*(*t*_1_)⋅*Q*(*t*_2_)⋅*Q*(*t*_3_)—the probability that the semantic variables of hidden layers *t*_1_, *t*_2_, *t*_3_ meet the translation needs.

The evaluation steps of the AE-based automatic TQA model for unreferenced English articles mainly include three steps. Firstly, the DL network is trained unsupervised from top to bottom. Each network layer is set as a Restricted Boltzmann Machine (RBM). The weights of each layer of the network are trained through a greedy learning algorithm, and the layered training is carried out from bottom to top. The first layer and other network layers are modeled respectively to obtain binary-binary RBM and Gaussian-Binary RBM. Hidden nodes and visible nodes are independent of each other in the RBM, and Eq (23) expresses their conditional probability distribution:

$$\theta_{1}=M(f_{j}+\varepsilon \sum \phi t_{1})$$ (23)

Then, Eq (24) manifests the JPD:

$$\theta_{2}=logistic\;\left(f_{j}+\sum_{j}\;\phi \frac{u_{j}}{\varepsilon }\right)$$ (24)

In Eq (24), *M*()—Gaussian density function; logistic—logical function; *f*_*j*_—bias of visual layer; *t*_1_—the number of nodes in the hidden layer is 1; *ε*—standard deviation; *ϕ*—weight.

Secondly, supervised overall fine-tuning is performed on the output layer according to the input bilingual word *V*_*E*_, *V*_*C*_.

Lastly, the bias and weight of each layer are obtained through supervised learning and unsupervised training, and a regression model that can output the characteristics of the translated article is implemented. Then, the translation quality is evaluated by using the proposed regression model. The proposed regression model is manifested in Eq (25):

$$\Omega =\phi \cdot V_{E}+\phi \cdot V_{C}$$ (25)

In Eq (25), Ω—automatic evaluation result of translation quality of unreferenced English articles; *ϕ*—weight.

RETRACTED

Further, the translation results of different software come from the average score of 30 English professors. The calculation method is given in Eq (26).


$$D=\frac{\sum_{i=1}^{30}\left(A_{i}\right)}{30}$$ (26)

In Eq (26), *A*_*i*_ represents the score given by the *i*th professor on the current evaluation index.

## Experimental results

### Model validity

This section takes the statements in a news website as the experimental data set based on the index evaluation standard of the *Translation Service Specification Part 1*: *Translation* compiled by China Translation Association. Then, the statement translation quality is automatically evaluated through the proposed regression model. Fig 5 details the statements on the news website:

**Fig 5:** Statement details on news website.

As shown in Fig 5, the translated news statements are evaluated by the proposed TQA model. The number of statements in the test set and training set of multiple languages is about 5,000. The translation details of various languages are shown in Fig 6:

**Fig 6:** Translation details.

When the effectiveness of the proposed model is evaluated, the difference between the actual situation and the automatic evaluation structure is set as the test index, and the test results of the proposed model are illustrated in Fig 7:

**Fig 7:** Evaluation results of the proposed model.

Comparing Figs 6 and 7 find that the difference between the evaluation results of correct sentences and the number of correctly translated sentences of the proposed model is 1. This is because there are differences in syntactic structures between different languages. Therefore, the translation quality evaluation of unreferenced English articles by the proposed model can meet the actual needs and, thus, can effectively evaluate the translation quality.

### Influence of translation sentence patterns on the evaluation performance of the proposed model

Further, the translated articles’ sentence structures are set as compound, interrogative, declarative, and special usage sentences. Then, the automatic evaluation results of the proposed TQA model are tested, as sketched in Fig 8:

**Fig 8:** Translation quality. a: declarative sentences, interrogative sentences, and compound sentences; b: special usage sentences.

As detailed in Fig 8, in the case of different sentence patterns translated, there is little difference between the actual translation of different languages and the evaluation results of the proposed model. Only the actual translation of special usage sentences differs from the evaluation results of the proposedly model, but the difference is only 1. The actual translation results of compound sentences, interrogative sentences, and declarative sentences are consistent with the evaluation results of the proposed model.

RETRACTED

### Influence of sentence numbers on the proposed TQA model’s performance

The actual translation quality and the evaluation result of the proposed TQA model for a given sentence are denoted as A1 and A2, respectively. The ratio between A2 and the correct evaluation result in A1 is the Bilingual Evaluation Understudy (BLEU) score. The BLEU can calculate the sum of sentences with translation errors in the test set to evaluate the performance of the proposed model. The results are given in Fig 9:

**Fig 9:** Proposed model evaluation performance affected by the number of sentences.

As plotted in Fig 9, when the number of sentences increases, the number of actual translation errors and the evaluation scores of the proposed TQA model increase, but the BLEU score is not significantly affected. When the number of sentences increases from 1,000 to 6,000, the BLEU score increases from 96 to 98, which shows that the proposed model has good performance.

### Practical application results

In this section, the proposed model is used to evaluate the translation quality of Baidu translation (A for short), Youdao translation (B), and Google translation (C) based on a translation text: *Presidential Election Season Brings Reality of U*.*S*. *Democracy into Spotlight*. The final translation results are shown in Fig 10 below:

**Fig 10:** Automatic evaluation results of the TQA model. a: vocabulary; b: discourse; c: grammar.

Fig 10 compares the grammar quality analysis results of Baidu translation, Youdao translation, and Google translation. From the vocabulary perspective, Fig 10A mainly analyzes the word meaning collocation, rhetoric, special terms, and dialect use of software translation. From the discourse perspective, Fig 10B mainly analyzes the software translation’s cohesion, coherence, intention, acceptability, information, context, and intertextuality. Apparently, software C has fewer errors in vocabulary and grammar than software A and B. However, its error rate in text translation is higher.

Next, the proposed model is compared with other literature methods: "Quality Evaluation of Machine Translation of Chinese Passive Voice—Taking Google translation and Youdao translation as an example" and "Research on Machine Translation Quality Evaluation Method Based on Questionnaire and Data Analysis." Fig 11 compares the evaluation accuracy of different methods to evaluate the proposed model’s effectiveness:

**Fig 11:** Comparison of model accuracy under different numbers of sentences.

RETRACTED

Fig 11 indicates that when the number of sentences is 1,000–6,000, compared with the methods in literature 1 and 2, the proposed model is obviously better than the other two models. The proposed model’s prediction accuracy is as high as 97%, and the stability is better, so it has a certain application value.

Further, to further evaluate the application value of the proposed model, Fig 12 compares the quality evaluation efficiency of the three models:

**Fig 12:** Comparison of model quality evaluation efficiency under different number of sentences.

As described in Fig 12, given 1,000–6,000 statements, the efficiency of the proposed TQA model for unreferenced English articles is significantly better than the other two literature methods, with the highest quality evaluation efficiency reaching over 95%. The accuracy of the translation quality evaluation can be guaranteed to a certain extent, indicating that the proposed model is highly feasible.

### Comparative analysis of algorithms

So far, BLEU is a widely used TQA method, whether it be the traditional MT statistic analysis or the popular NN-based MT evaluation or training. Although many automatic TQA methods have received higher manual evaluation correlation than BLEU, BLEU remains the most widespread TQA. Generally, MT systems are trained by the Minimum Error Rate Training (MERT) based on multi-feature representation. MERT optimizes the MT system by minimizing the translation error rate. Specifically, the feature weight is optimized on the development set to gain the optimal automatic evaluation index. Common evaluation indexes include BLEU, Testing Error Rate (TER), and METEOR. In order to control the possible impact of each system module, the same MT system is trained and used in the subsequent experiment. The MT system chooses a Translation Model (TM) trained from the Linguistic Data Consortium (LDC)-provided bilingual corpus. This corpus included LDC2002E18, LDC2003E14, LDC2004E12, LDC2004T08, LDC2005T10, and LDC2007T09 data sets, totaling 8.3 million pairs of Chinese-English translation data. The Chinese part uses the ICT-CLAS word segmentation tool. The language model (LM) is trained by a monolingual corpus composed of the Xinhua and Gigaword corpus. The order of LM is 5. The development set uses the MT03 dataset with multiple reference translations. There are three test sets: MT02, MT04, and MT05, all containing multiple reference translations.

RETRACTED

Experimental Step 1 analyzes the performance of the BLEU+MERT MT system. The default experimental configuration and quality evaluation method are used in the experiment. The experimental results are drawn in Fig 13:

**Fig 13:** Comparison of experimental results.

After being trained by BLEU, TER, and METEOR, the TER-trained MT system has the translation missing issue, and the translated sentences are too short. Simultaneously, the BLEU-trained system also has a small amount of missing translation but shows a much-improved translation quality than the TER-trained system. By comparison, the METEOR system over translates and generates long redundant sentences. Overall, the BLEU-trained MT system presented a stable performance in all evaluation indexes. The findings reveal why the BLEU evaluation indexes are chosen in the present work.

### Conclusions

MT evaluation is divided into two directions: one evaluates the MTS referring to prior human translations, and the other evaluates the MTS without reference to artificial translation. Most of the work focuses on the first task. In the past decade, researchers have done a lot of work on the second task. Indisputably, a suitable evaluation method helps improve the performance of the MTS. Therefore, the rapid development of MT drives the continuous development of evaluation technology. At the same time, more and more evaluation activities also promote the constant development of translation evaluation technology. In return, competitive evaluation activities promote MT performance to a certain extent.

Thereupon, this paper proposes an unreferenced English articles-oriented automatic TQA model based on SAE under the background of DL. Then, the DL-based automatic translation language-oriented information extraction method employs AE in the bilingual words’ unsupervised learning stage. It reconstructs the language vector features of the sample unreferenced English articles to be translated. Afterward, it imports the translation information of unreferenced English articles into bilingual words and optimizes the extraction effect of language vector features. The translation language vector feature is introduced into the proposed DL-based automatic TQA model. The experimental results corroborate that the difference between the evaluation results of correct sentences and the number of correctly translated sentences is 1, and the accuracy of the evaluation results is high. When the number of sentences increases, the number of actual translation errors and the evaluation scores of the model increase, but the BLEU is not significantly affected. When the number of sentences increases from 1,000 to 6,000, the BLEU increases from 96 to 98, which shows that the proposed TQA model has good performance.

RETRACTED

However, there are still some problems with the research content. Due to the complexity of translation activities, there are still some difficulties in the comprehensive evaluation of translation. At present, there is no definite conclusion on the evaluation criteria of translation, and there are differences in evaluation parameters and weights, so it isn’t easy to propose an evaluation model that meets all translation requirements and has strong operability. Therefore, to promote the development of automatic evaluation technology, future work will focus on the above problems.

## Supporting information

S1 Data (RAR)

## References

[1] OrganM. Translation Technology in English Studies Within the System of Higher Education in Poland. International Journal of English Linguistics. 2021; 11(4): 1.

[2] TaoY, WangH. Translation technology teaching: views and visions. The Interpreter and translator trainer. 2020; 14(4): 478–479.

[3] LiM, ZhouC, Henriksen LB. A Socio-technical-cultural System Perspective to Rethinking Translation Technology in Intercultural Communication. Communication & Language at Work. 2020; 7(1): 100–110.

[4] FengH. The Future of Translation Technology–Towards a world without Babel. Terminology. 2018; 24(2): 295–299.

[5] Wadyka-Leittretter AM. The Future of Translation Technology. Towards a World without Babel. (Review). The Journal of Specialised Translation. 2018; 29: 255–256.

[6] HouZ. The Metaphor Processing and Translation Skills of Computer Technology in English Language Translation. Journal of Physics Conference Series. 2021; 1744(4): 042125.

[7] Han X, Zhu J, Zhang F, He Y, Zhong H. Research on Key Technology of Integral Translation and Rotation of the Large-Diameter Shield and Steel Sleeve in the Underwater Tunnel of the Karnaphuli River, Bangladesh. IOP Conference Series: Earth and Environmental Science. 2021; 783(1): 012117.

[8] ShortenC, Khoshgoftaar TM, FurhtB. Deep Learning applications for COVID-19. Journal of Big Data, 2021, 8(1): 1–543345718110.1186/s40537-020-00392-9PMC7797891

[9] YangT, FanH. Application of Computer Technology in English Translation. Journal of Physics Conference Series. 2020; 1575: 012029.

[10] AbdiH. Translation and Technology: Investigating the Employment of Computer-aided Translation (CAT) Tools among Iranian Freelance Translators. Theory and Practice in Language Studies. 2020; 10(7): 811.

[11] Xie SX, Yu ZC, Lv ZH. Multi-disease prediction based on deep learning: a survey. Computer Modeling in Engineering & Sciences. 2021.

[12] Lv ZH, Chen DL, CaoB, Song HB, Lv HB. Secure Deep Learning in Defense in Deep-Learning-as-a-Service Computing Systems in Digital Twins. IEEE Transactions on Computers. 2021.

RETRACTED

[13] LiY, Zhao JL, Lv ZH, Li JH. Medical Image Fusion Method by Deep Learning. International Journal of Cognitive Computing in Engineering. 2021.

[14] ZaidiI, ChtourouM, DjemelM. Robust Neural Control of Discrete Time Uncertain Nonlinear Systems Using Sliding Mode Backpropagation Training Algorithm. International Journal of Automation and Computing. 2019; 16(02): 87–99.

[15] Lin JW, Chao CT, Chiou JS. Backpropagation neural network as earthquake early warning tool using a new modified elementary Levenberg–Marquardt Algorithm to minimise back-propagation errors. Geoscientific Instrumentation Methods & Data Systems. 2018; 7(3): 235–243.

[16] KrestinskayaO, Salama KN, James AP. Learning in Memristive Neural Network Architectures Using Analog Backpropagation Circuits. IEEE Transactions on Circuits and Systems I: Regular Papers. 2018; 66: 719–732.

[17] Kshirsagar PR, ManoharanH, TirthV, NavedM, Sharma AK. Automation Monitoring With Sensors For Detecting Covid Using Backpropagation Algorithm. KSII Transactions on Internet and Information Systems. 2021; 15(7): 2414–2433.

[18] WatabeM, ShibaK, Chen CC, SogabeM, SogabeT. Quantum Circuit Learning with Error Backpropagation Algorithm and Experimental Implementation. Quantum Reports. 2021; 3(2): 333–349.

[19] Lu HW, Yu XP, Wang SQ, Liu YY, Chen JM. A digital background calibration scheme for non-linearity of SAR ADC using back-propagation algorithm. Microelectronics Journal. 2021; 114(104): 105113.

[20] ChenJ, RongY, ZhuQ, ChandraB, ZhongH. A generalized minimal residual based iterative back propagation algorithm for polynomial nonlinear models. Systems & Control Letters. 2021; 153(2): 104966.

[21] MaX, GuanY, MaoR, ZhengS, WeiQ. Modeling of lead removal by living Scenedesmus obliquus using back-propagation (BP) neural network algorithm. Environmental Technology & Innovation. 2021; 22(s1-2): 101410.

[22] YangF, MaB, WangJ, GaoH, LiuZ. Target Detection of UAV Aerial Image Based on Rotational Invariant Depth Denoising Automatic Encoder. Xibei Gongye Daxue Xuebao/Journal of Northwestern Polytechnical University. 2020; 38(6): 1345–1351.

[23] FanZ, LiC, ChenY, WeiJ, Mascio PD. Automatic Crack Detection on Road Pavements Using Encoder-Decoder Architecture. Materials. 2020; 13(13): 2960. doi: 10.3390/ma13132960 32630713PMC7372440

[24] ChengC, ShangZ, ShenZ. Automatic delamination segmentation for bridge deck based on encoder-decoder deep learning through UAV-based thermography. NDT & E International. 2020; 116: 102341.

[25] PietroC, AntonellaB, GuidoB, AlfonsoM. Stacked sparse autoencoder networks and statistical shape models for automatic staging of distal femur trochlear dysplasia. International Journal of Medical Robotics and Computer Assisted Surgery. 2018; 14: e1947. doi: 10.1002/rcs.1947 30073759

RETRACTED

[26] MeiS, WangY, WenG. Automatic Fabric Defect Detection with a Multi-Scale Convolutional Denoising Autoencoder Network Model. Sensors. 2018; 18(4): 1064. doi: 10.3390/s18041064 29614813PMC5948749

[27] ZhaiJ, ShiH, WangM, SunZ, XingJ. An Encrypted Traffic Identification Scheme Based on the Multilevel Structure and Variational Automatic Encoder. Security and Communication Networks. 2020; 2020(11): 1–10.

[28] ShinJ, Lee WK, KimY, Han HJ, Lee JH. Research on the Decoder Attention Structure of Multi-encoder Transformer-based Automatic Post-Editing Model. KIISE Transactions on Computing Practices. 2020; 26(8): 367–372.

[29] J KwakSung Y. Automatic 3D Landmark Extraction System Based on an Encoder–Decoder Using Fusion of Vision and LiDAR. Remote Sensing. 2020; 12(7): 1142.

[30] JwaH, OhD, ParkK, Kang JM, LimH. exBAKE: Automatic Fake News Detection Model Based on Bidirectional Encoder Representations from Transformers (BERT). Applied Sciences. 2019; 9(19): 4062.

[31] WangZ, JoshiS, Savel’EvS, SongW, MidyaR, LiY, et al. Fully memristive neural networks for pattern classification with unsupervised learning. Nature Electronics. 2018; 1(2): 137–145.

[32] XiJ, LiA, WangM. A novel unsupervised learning model for detecting driver genes from pan-cancer data through matrix tri-factorization framework with pairwise similarities constraints. Neurocomputing. 2018; 296(JUN.28): 64–73.

[33] HuebnerD, VerhoevenT, Mueller KR, Kindermans PJ, TangermannM. Unsupervised Learning for Brain-Computer Interfaces Based on Event-Related Potentials: Review and Online Comparison [Research Frontier]. IEEE Computational Intelligence Magazine. 2018; 13(2): 66–77.

[34] Biaz BM, Ferreira VH, Fortes MZ, Lopes TT, LimaG. Islanding Detection in Distributed Generation using Unsupervised Learning Techniques. IEEE Latin America Transactions. 2018; 16(1): 118–125.

[35] Chandra GM, ReddyG. Framework for Contextual Outlier Identification using Multivariate Analysis approach and Unsupervised Learning. International Journal of Electrical & Computer Engineering. 2018; 81(2): 1092–1101.

